# Severity Assessment of COVID-19 Using a CT-Based Radiomics Model

**DOI:** 10.1155/2021/2263469

**Published:** 2021-09-27

**Authors:** Zhigao Xu, Lili Zhao, Guoqiang Yang, Ying Ren, Jinlong Wu, Yuwei Xia, Xuhong Yang, Milan Cao, Guojiang Zhang, Taisong Peng, Jiafeng Zhao, Hui Yang, Jinfeng Hu, Jiangfeng Du

**Affiliations:** ^1^College of Medical Imaging, Shanxi Medical University, Taiyuan, 030001 Shanxi Province, China; ^2^Department of Radiology, The Third People's Hospital of Datong, Datong, 037008 Shanxi Province, China; ^3^Department of Radiology, First Hospital of Shanxi Medical University, Taiyuan, 030001 Shanxi Province, China; ^4^Department of Materials Science and Engineering, Henan University of Technology, Zhengzhou, 450001 Henan Province, China; ^5^Huiying Medical Technology Co., Ltd, Room A206, B2, Dongsheng Science and Technology Park, Haidian District, Beijing City, 100192, China; ^6^Department of Science and Education, The Third People's Hospital of Datong, Datong, 037008 Shanxi Province, China; ^7^Department of Radiology, The Second People's Hospital of Datong, Datong, 037005 Shanxi Province, China; ^8^Department of Rehabilitation Medicine, Xiantao First People's Hospital, Xiantao, 433000 Hubei Province, China

## Abstract

The coronavirus disease of 2019 (COVID-19) has evolved into a worldwide pandemic. Although CT is sensitive in detecting lesions and assessing their severity, these works mainly depend on radiologists' subjective judgment, which is inefficient in case of a large-scale outbreak. This work focuses on developing a CT-based radiomics model to assess whether COVID-19 patients are in the early, progressive, severe, or absorption stages of the disease. We retrospectively analyzed the CT images of 284 COVID-19 patients. All of the patients were divided into four groups (0-3): early (*n* = 75), progressive (*n* = 58), severe (*n* = 75), and absorption (*n* = 76) groups, according to the progression of the disease and the CT features. Meanwhile, they were split randomly to training and test datasets with the fixed ratio of 7 : 3 in each category. Thirty-eight radiomic features were nominated from 1688 radiomic features after using select *K*-best method and the ElasticNet algorithm. On this basis, a support vector machine (SVM) classifier was trained to build this model. Receiver operating characteristic (ROC) curves were generated to determine the diagnostic performance of various models. The precision, recall, and *f*_1_-score of the classification model of macro- and microaverage were 0.82, 0.82, 0.81, 0.81, 0.81, and 0.81 for the training dataset and 0.75, 0.73, 0.73, 0.72, 0.72, and 0.72 for the test dataset. The AUCs for groups 0, 1, 2, and 3 on the training dataset were 0.99, 0.97, 0.96, and 0.93, and the microaverage AUC was 0.97 with a macroaverage AUC of 0.97. On the test dataset, AUCs for each group were 0.97, 0.86, 0.83, and 0.89 and the microaverage AUC was 0.89 with a macroaverage AUC of 0.90. The CT-based radiomics model proved efficacious in assessing the severity of COVID-19.

## 1. Introduction

The outbreak of coronavirus disease 2019 (COVID-19), which began in December 2019, is a severe acute respiratory syndrome coronavirus 2 (SARS-CoV-2) infection. The World Health Organization (WHO) has declared COVID-19 a global pandemic, and by 6 August 2021, there have been 200,840,180 confirmed cases of COVID-19, including 4,265,903 deaths, reported to the WHO [1]. Nucleic acid testing (NAT) of the reverse transcription polymerase chain reaction (RT-PCR) is currently the most reliable diagnostic method for COVID-19, but chest computed tomography (CT) is recognized as an important tool for severity assessment, as well as an important complementary diagnostic technique. Therefore, chest CT has become an indispensable tool in the screening and severity assessment of COVID-19.

When the number of infected people is small and the number of doctors is sufficient, it is feasible to assess the severity of such patients manually; however, in case of a large-scale outbreak, there may be too few radiologists. Therefore, the development of automated and reproducible analysis methods to extract more information from image-based features is a requirement. Radiomics—the high-throughput extraction of large amounts of image features from radiographic images—addresses this problem and is one of the approaches that hold great promise [2]. Researchers have proposed the use of radiomic features to quantify various tumor phenotypes on medical images, to describe this heterogeneity and furthermore, and utilize these features as predictors of genetics and clinical outcomes [3]. For the diagnosis of COVID-19 based on GGO lesions, a CT-based radiomics model could be a promising supplementary tool for improving specificity for COVID-19 in a population confounded by ground glass opacity changes from other etiologies. Furthermore, the assistance afforded by application of artificial intelligence has improved radiologists' performance in distinguishing coronavirus disease 2019 pneumonia from noncoronavirus disease 2019 pneumonia at chest CT.

Therefore, to relieve pressure on radiologists when evaluating the severity of COVID-19 and to avoid mistakes under fatigue, the present research establishes a radiomics model by evaluating the relationship between CT staging and CT-based radiomics characteristics of COVID-19.

## 2. Materials and Methods

### 2.1. Patient Population and Ethical Approval

Our institutional review board (IRB) waived written informed consent for this retrospective study, which evaluated deidentified data and brought no potential risk to patients. To avert any potential breach of confidentiality, no link between the patients and the researchers was available.

Patient data were collected from the First People's Hospital of Xiantao of China, during the period between February 2020 and June 2020. The inclusion criterion of COVID-19 was conformity to the Diagnosis and Treatment of COVID-19 (revised edition of the provisional 7^th^ edition) which forms the guidelines for the National Health Commission of the People's Republic of China [4]. We included patients having a history of contact in epidemic areas or with known patients: these patients had been confirmed as COVID-19 cases by polymerase chain reaction (PCR). Meanwhile, the inclusion criteria also included the following: (1) patients have received CT examination, and the CT images can be obtained; (2) there were no other chest diseases or history of chest surgery in these patients before CT examination; and (3) their clinical data are complete and comprehensive. The exclusion criteria include the following: (1) the quality of CT images is so poor that they cannot be used for analysis, and (2) chest CT shows other chest diseases, such as tuberculosis and lung cancer. Clinical information and chest CT data of 303 consecutive COVID-19 patients with COVID-19 were collected.

For this study, 284 COVID-19 patients were enrolled. There were 123 males and 161 females, aged from 1 to 91 years old, with a mean average age of 55.50 ± 14.97 y. In the training set, there were 89 males and 108 females, with a mean average age of 54.56 ± 15.47 y (ranging from ages of 1 to 91 y); in the test set, there were 34 males and 53 females, with a mean average age of 57.61 ± 13.61 y (ranging from ages of 29 to 89 y).

### 2.2. CT Examination

The GE Optima 660 and GE Optima 540 spiral CT scanners were used. Patients adopted a supine position, and scanning was performed at the end of inspiration using the conventional dose. For each patient, the scanning range was from the apex of the lung to the costophrenic angle, the slice thickness was 5 mm, the tube voltage was 120 kV, and the tube current was 100 mA. All imaging data were reconstructed by using a medium-sharp reconstruction algorithm with a thickness of 1.25 mm.

### 2.3. Marking of CT Images

Original CT images, which were exported in DICOM format from CT scanners, were uploaded to Radcloud (Huiying Medical Technology Co., Ltd, Beijing, China). Subsequently, CT features of COVID-19 patients were investigated. The location, morphology, distribution, extent, density, and internal structure of the lesions were observed to identify features such as thickened lobular septum and central nodules of the lung lobules. The relationships between lesions and bronchial blood vessels, the condition of stripe signs, and the presence of solid component signs were determined. Morphological changes and imaging signs were observed in patients with dynamic follow-up.

For each patient, the severity of COVID-19 was determined following both the guidelines in 2019-nCoV (Trial Version 7) issued by the China National Health Commission and the guidelines for medical imaging in auxiliary diagnosis of coronavirus disease 2019 issued by the Chinese Research Hospital Association Radiology Committee on Infectious and Inflammatory Disease, et al. [4, 5]. COVID-19 is classified into four stages: mild, moderate, severe, and resorption stages, based on the severity thereof: (1) early stage: focal ground-glass opacity (GGO) was not distributed across segments, but multiple lesions may occur; (2) advanced stage: the lesions were distributed across segments and had a large range of GGO, including the paving-stone sign and mixed GGO and solid component signs. There were also solid component signs, regardless of the size of the range; (3) severe stage: it developed from the advanced stage, and the lesion area had increased significantly based on previous examination. The CT manifestation was evinced by the presence of “butterfly sign” and even “white lung”; and (4) resorption stage (or recovery stage): the main manifestation was the narrowed lesion range and the lightened density based on data from the previous stage, and the characteristic stripe sign appeared.

The segmented images marked by experts were used as the standard to evaluate the collected thin-layer CT images. Two radiologists, each with at least five years of chest-imaging experience, manually outlined the ROI using the labelling tool in the Radcloud platform. They considered the distribution and image features of disease foci in COVID-19 (Figures 1–4). In the event of disagreement between the two primary radiological interpretations, a third experienced thoracic radiologist with 16 years of experience adjudicated in reaching a final decision.

### 2.4. Radiomic Feature Extraction

After image preprocessing, 1688 radiomic features were extracted for each subject using the PyRadiomics v3.0 (open source software), including original features and features (original features except shape features) as transformed by logarithm, wavelet (LLL, LLH, LHL, LHH, HLL, HLH, HHH, and HHL), exponent, gradient, square, square root, and local binary pattern applied in 2D and 3D. Among 107 original features, 14 were related to shape features, 18 first-order, and 24 GLCM (grey-level cooccurrence matrix), 14 GLDM (grey-level dependence matrix), 16 GLRLM (grey-level run length matrix), 16 GLSZM (grey-level size zone matrix), and five NGTDM (neighboring grey-tone difference matrix) features. First-order statistics describe the distribution of voxel intensities within the image region defined by the mask through commonly used basic metrics. GLCM describes the second-order joint probability function of an image region constrained by the mask. GLDM quantifies grey-level dependencies in an image. GLRLM quantifies grey-level runs, which are defined as the length in number of pixels, of consecutive pixels that have the same grey-level value. GLSZM quantifies grey-level zones in an image. A grey-level zone is defined as the number of connected voxels that share the same grey-level intensity. NGTDM quantifies the difference between a grey-value and the mean average grey value of its neighbors within a preset distance. Detailed information about these features is available in the documentation supplied with the PyRadiomics software.

### 2.5. Feature Selection and Model Building

To verify the credibility of the manual segmentation between the two radiologists, the CT scans of 10 patients were randomly selected and segmented by the two radiologists for double-blind interpretation. Interclass correlation coefficients (ICC), which can be used to assess the interobserver reproducibility of ROIs delineated, can be obtained from the following equation:

(1) $$\begin{array}{c} \text{ICC}=\frac{\left({\text{MS}}_{\text{R}}-{\text{MS}}_{\text{E}}\right)}{{\text{MS}}_{\text{R}}+\left(\left({\text{MS}}_{\text{C}}-{\text{MS}}_{\text{E}}\right)/n\right)}, \end{array}$$

where MS_R_ represents mean square for rows; MS_C_ is mean square for columns; MS_E_ denotes mean square for error; and *n* is the number of subjects. The value of ICC was greater than 0.75.

After feature extraction, 70% of the dataset was randomly assigned to the training set and for all cases, features were normalized to the normal distribution by mean and variance scaling. The trained SVM classifier was evaluated on the test dataset while the training and feature selection was conducted only on the training data. *K*-best was applied to select the most significantly relevant feature set with threshold of 0.05. To avoid overfitting caused by the radiomic features being larger than the sample size, ElasticNet, a regularized, generalized model, linearly combines the *L*_1_ and *L*_2_ penalties of the least absolute shrinkage and selection operator and ridge methods to realize a built-in feature weighting mechanism, making an appropriate balance between model generalization and diagnostic performance. The model was trained with 10-fold cross-validation to attain the optimal *α*-value. Following the optimal *α*-value, an optimal simplified feature set was determined. An SVM classifier was built to distinguish among the four COVID-19 groups based on final reduced imaging radiomic features. The receiver operating characteristic (ROC) curve was plotted as a classifier of each group, and the area under the curve (AUC) measure was applied to evaluate model performance. The 95% confidence level was assessed on the variation of the AUC. Micro- and macroaverage AUC, precision, recall, and *f*_1_-score were also calculated to assess model performance for multiclass classification.

## 3. Results

### 3.1. The Radiomics Workflow

The radiomics workflow is illustrated in Figure 5. In this study, 284 patients were retrospectively included to investigate the validity of radiomics-based classification with 75, 58, 75, and 76 cases, respectively, for groups 0, 1, 2, and 3 (early stage, progressive stage, severe stage, and absorptive stage). The dataset was split at random to form training and test datasets with a fixed ratio of 7 : 3 in each category, resulting in 197 (52 cases in group 0, 40 in group 1, 52 in group 2, and 53 in group 3) for the training dataset and 87 cases for the test dataset.

### 3.2. Radiomic Features

Of all the radiomic features extracted, the median ICC was 0.885; 1011 of 1688 features (59.9%) were robust, with ICC > 0.75. Then, 38 radiomic features were nominated from 1688 radiomic features after using select *K*-best method and the ElasticNet algorithm (Figure 6 and Table 1). The 38 features contain four first-order features, two shape features, nine grey-level cooccurrence matrix (GLCM) features, 10 grey-level dependence matrix (GLDM) features, five grey-level run length matrix (GLRLM) features, six neighboring grey-tone difference matrix (NGTDM) features, and two grey-level size zone matrix (GLSZM) features.

### 3.3. Model Classification Performance

An SVM classifier was trained based on optimal feature set on training dataset. The precision, recall, and *f*_1_-score of the classification model for the macroaverage and microaverage were 0.82, 0.82, 0.81, 0.81, 0.81, and 0.81 for the training dataset and 0.75, 0.73, 0.73, 0.72, 0.72, and 0.72 for the test dataset. The AUCs for groups 0, 1, 2, and 3 on the training dataset were 0.99, 0.97, 0.96, and 0.93, and the microaverage AUC was 0.97 with a macroaverage AUC of 0.97 (Figure 7(a)). On the test dataset, AUCs for each group were 0.97, 0.86, 0.83, and 0.89 and the microaverage AUC was 0.89 with a macroaverage AUC of 0.90 (Figure 7(b)).

## 4. Discussion

Assessing pulmonary lesions using computed tomography (CT) images is of significance to the severity diagnosis and treatment of coronavirus disease 2019- (COVID-19-) infected patients. Such assessment mainly depends on the subjective judgment of radiologists, which is inefficient and presents difficulties for those with low levels of experience, especially in primary or community hospitals [6–8]. In this study, we uncover some of the radiomic features that contribute to evaluation of the severity of COVID-19 patients. A radiomics model aiming at assessing automatically the severity of COVID-19 was demonstrated, with favorable predictive accuracy, achieving an average AUC performance of 0.97 on a training dataset and 0.90 on a test dataset. Prediction outputs generated from our radiomics model further augmented human expert performance. More importantly, the model is expected to relieve the workload of radiologists and provide rapid, accurate severity assessments for COVID-19 patients.

Studies have found that the development of COVID-19 pneumonia is usually related to the increase in the number and size of GGO lesions [9]. In the early stage, there will be multiple small plaque shadows and interstitial changes in the lungs. CT in the middle stage of the disease shows an increase in the number and size of GGO, and GGO gradually transforms into multifocal consolidation; about 10 days after the onset of symptoms, the consolidation range often reaches its maximum, and it is transformed into fibrosis in the late stage [10–12]. Therefore, chest CT findings tend to be used as one of clinical manifestations in the confirmation of the diagnosis of COVID-19 infection [4]. Many clinical studies have investigated the CT imaging signs related to COVID-19 infection such as GGO, GGO with lung consolidation, interlobular septal thickening, and pulmonary fibrosis for patients at different stages and severity [13–15].

According to the time of onset, clinical manifestations, lesion range, and CT manifestations, COVID-19 can be roughly divided into four stages: early stage, advanced stage, severe stage, and resorption stage (recovery stage) [4, 5]. In this study, 284 patients were retrospectively graded as early stage with 75 cases, progressive stage with 58 cases, severe stage with 75 cases, and absorptive stage with 76 cases. Early-stage COVID-19 manifested as single or multiple nodules with mixed GGO as the main part, and the boundaries were blurred with a “halo sign,” and some showed a “thickened blood vessel” sign. Compared with the early-stage CT findings, the lesion range of progressive-stage COVID-19 was further expanded, the density increased, and fusion or mass-like consolidation appeared. In severe cases, diffuse lesions of both lungs are often present. The CT image showed a large patchy or fusion-like consolidation with symmetrical distribution across both lungs, showing a “butterfly sign” or “upside-down butterfly sign” and even presenting with “white lung.” The COVID-19 resorption stage (recovery stage) was manifested as the density of lesions decreased, and it is gradually completely absorbed, or GGO is completely resorbed, leaving a few stripes or small patchy consolidation signs, or consolidations are gradually replaced by GGO with stripes. Although chest CT has high sensitivity when identifying COVID-19 infection and evaluating its severity, the result mainly depends on the subjective judgment of the radiologist(s) and the work is time-consuming [16, 17].

In this article, an ElasticNet radiomics model was exploited and investigated to evaluate the severity of COVID-19 patients. Ground-glass opacities and consolidation are the most relevant imaging features in COVID-19 pneumonia [17], which were identified by chest CT with high sensitivity. A radiomics model based on machine learning can detect minute changes in the VOIs which are difficult to see with the naked eye, let alone estimate the size thereof; thus, the radiological features hidden in GGO lesions are extracted and quantified: CT-based radiomics characteristics such as the degree and density of GGO can divide patients with COVID-19 pneumonia into different development stages [18, 19].

The radiomics model of COVID-19 studies based on CT images involves predominantly of diagnostic and prognostic value; a majority of the recently published studies focus on the diagnosis and differentiation of COVID-19 such as those using UNet for automated detection of GGO areas [20, 21] and differentiation of COVID-19 pneumonia from other viral pneumonia using radiomics or deep-learning methods [22–24]. However, to the best of our knowledge, there have been few studies on the validity of CT for assisting decision-making in the management of COVID-19 with regard to stratification of disease severity and prediction of clinical outcomes [18, 25]. Additionally, few studies have focused on the use of a radiomics model to assess the severity of COVID-19: one study classifying two types of COVID-19 severity (nonsevere and severe) instead of four types was undertaken to assess the relevance of CT image features [26]. Research by Cai et al. stratifies the severity into moderate, severe, and critical groups with AUCs greater than 0.925 [20]. In the present study, we collected more CT image data from COVID-19 patients; all patients were divided into four developmental stages: early stage, advanced stage, severe stage, and prognosis stage according to the essence of lung GGO lesions; then, we stratified the severity of the disease by CT quantification.

Using a select *K-*best method, 38 radiological characteristics were nominated from 1688 radiomic features in our study, which reflected intrinsic information such as lesion intensity and textural features that cannot otherwise be detected by radiologists [27]. For example, first-order features mainly reflect the internal texture of lesions; wavelet features mainly reflect the change of time domain and frequency domain information within the lesion [28]. Among the 38 features, six first-order features, 30 texture features, and two shape features comprised the optimal feature set, indicating different feature dimensions to be considered during the staging of COVID-19. The five most relevant features are logarithm_first-order_Skewness, wavelet-HHH_first-order_10Percentile, original_shape_Sphericity, wavelet-HLH_gldm_SmallDependenceEmphasis, and wavelet-LLL_glcm_Inverse Variance, four of which are high-order features transformed by different filters. Logarithm_first-order_Skewness measured the asymmetry of the distribution of values about the mean value, wavelet-HHH_first-order_10Percentile denoted the 10^th^ percentile of the image, original_shape_Sphericity equated the roundness of the shape of the VOI to a sphere, and wavelet-HLH_gldm_SmallDependenceEmphasis assessed the distribution of small dependencies. In our research, four types of severity groups of COVID-19 were distinguished by SVM classifier; then, the ROC curve of each group was plotted. Finally, the ElasticNet radiomics model shows favorable predictive accuracy, achieving an average AUC performance of 0.97 on the training dataset and one of 0.90 on the test dataset, indicating the strong efficacy of the proposed CT-based radiomics model in assessing the severity of COVID-19 disease.

## 5. Conclusions

A CT-based radiomics model was provided that can be used to assess the severity of COVID-19, which can help radiologists undertake rapid diagnosis, especially useful when the medical system is overloaded.

## 6. Limitations

Our research has several limitations. First of all, this was a retrospective study; we divided COVID-19 patients into four severity levels based on the CT imaging manifestations of COVID-19 patients, such as the degree of GGO lesions, without combining specific clinical symptoms and other factors: some studies have shown that the CT manifestations of COVID-19 may vary with age; elderly patients predominantly present with combined features such as opacity, while young patients present predominantly GGO [9], which may lead to inaccurate demarcation and introduce selection bias. Besides, our research lacks multicenter verification: use of only a single device and model may limit the popularization and application of the results.

## Figures and Tables

**Figure 1:** A case of confirmed mild COVID-19. A 33-year-old female presented with a 2-day history of fever and cough. (a) CT imaging revealed diffuse pure GGO with distribution in the left lower lobe. The area of the lesions was delineated on the axial. (b) The reconstructed images.

**Figure 2:** A case of confirmed mild COVID-19. A 63-year-old male presented with a 5-day history of fever, cough, and mild dyspnea. (a) CT imaging revealed pure GGO with distribution in the left lower lobe. The area of the lesions was delineated on the axial. (b) The reconstructed images.

**Figure 3:** A case of confirmed severe COVID-19. A 45-year-old male presented with a 12-day history of fever, cough with expectoration, and mild dyspnea. (a). CT imaging revealed multiple consolidation with symmetric distribution in both lungs. The area of the lesions was delineated on the axial. (b) The reconstructed images.

**Figure 4:** A case of confirmed COVID-19 of the resorption stage. A 63-year-old male presented with a 15-day history of fever and cough. (a). CT imaging revealed pure GGO with reticular distributed in the right lower lobe. The area of the lesions was delineated on the axial. (b) The reconstructed images.

**Figure 5:** Flowchart through the study.

**Figure 6:** ElasticNet algorithm for feature selection. The first (a) shows coefficient profiles along the full path of possible values for radiomic features. The MSE path (b) indicates that the dotted vertical line was plotted at the value selected using 10-fold cross-validation in (a). The coefficients in the ElasticNet model (c) resulted in 38 features based on selected optimal values.

**Figure 7:** ROC curves of the SVM classifier on the training set (a) and test set (b).

**Table 1:** Description of the selected radiomic features and their associated feature types and filters.

Radiomic features	Associated_filters	Types
Logarithm_firstorder_Skewness	Logarithm	First order
Logarithm_firstorder_Kurtosis	Logarithm	First order
Llogarithm_glcm_InverseVariance	Logarithm	GLCM
Original_shape_Sphericity	Original	SHAPE
Exponential_gldm_DependenceEntropy	Exponential	GLDM
Gradient_gldm_LowGrayLevelEmphasis	Gradient	GLDM
Gradient_glrlm_ShortRunLowGrayLevelEmphasis	Gradient	GLRLM
Original_shape_Maximum2DDiameterSlice	Original	SHAPE
Exponential_glcm_Correlation	Exponential	GLCM
Wavelet-HLL_ngtdm_Complexity	Wavelet-HLL	NGTDM
Gradient_ngtdm_Complexity	Gradient	NGTDM
Wavelet-LHH_gldm_GrayLevelNonUniformity	Wavelet-LHH	GLDM
Squareroot_glcm_Contrast	Squareroot	GLCM
lbp-2D_gldm_DependenceEntropy	lbp-2D	GLDM
lbp-3D-m1_gldm_DependenceEntropy	lbp-3D-m1	GLDM
Original_ngtdm_Busyness	Original	NGTDM
lbp-3D-m2_gldm_DependenceEntropy	lbp-3D-m2	GLDM
lbp-3D-k_gldm_HighGrayLevelEmphasis	lbp-3D-k	GLDM
lbp-3D-k_gldm_LowGrayLevelEmphasis	lbp-3D-k	GLDM
lbp-3D-k_glcm_MaximumProbability	lbp-3D-k	GLCM
lbp-3D-k_glrlm_ShortRunEmphasis	lbp-3D-k	GLRLM
lbp-3D-k_glcm_Autocorrelation	lbp-3D-k	GLCM
lbp-3D-k_ngtdm_Contrast	lbp-3D-k	NGTDM
lbp-3D-k_glcm_ClusterProminence	lbp-3D-k	GLCM
Wavelet-LLL_glcm_InverseVariance	Wavelet-LLL	GLCM
lbp-3D-k_glrlm_ShortRunHighGrayLevelEmphasis	lbp-3D-k	GLRLM
Wavelet-LLL_glcm_MCC	Wavelet-LLL	GLCM
Wavelet-HLH_glszm_ZonePercentage	Wavelet-HLH	GLSZM
Wavelet-HLH_gldm_SmallDependenceEmphasis	Wavelet-HLH	GLDM
Wavelet-HLH_glcm_MCC	Wavelet-HLH	GLCM
Wavelet-HLH_glszm_SmallAreaEmphasis	Wavelet-HLH	GLSZM
Wavelet-LLH_firstorder_Skewness	Wavelet-LLH	First order
Wavelet-HHH_firstorder_10Percentile	Wavelet-HHH	First order
Wavelet-LLL_gldm_DependenceVariance	Wavelet-LLL	GLDM
lbp-3D-k_firstorder_Skewness	lbp-3D-k	First order
Wavelet-HHL_ngtdm_Complexity	Wavelet-HHL	NGTDM
Wavelet-LLH_firstorder_Mean	Wavelet-LLH	First order
Wavelet-LHH_ngtdm_Busyness	Wavelet-LHH	NGTDM

GLCM: grey-level cooccurrence matrix; GLRLM: grey-level run length matrix; GLSZM: grey-level size zone matrix; NGTDM: neighboring grey-tone difference matrix; GLDM: grey-level dependence matrix.

## Data Availability

The supporting data are available in Radcloud (Huiying Medical Technology Co., Ltd, Beijing, China) and can be made available upon reasonable request. The datasets generated during this study are available from the corresponding author upon reasonable request.
